# Construction of Smart Higher Education Teaching Resources Using Data Analysis Technology in Unbalanced Data Environment

**DOI:** 10.1155/2022/2130623

**Published:** 2022-09-20

**Authors:** Yuting Luo

**Affiliations:** Informatization Center, Nantong University, Nantong Jiangsu 226019, China

## Abstract

The difficulty in gathering teaching resources presents challenges in the process of developing instructional materials for smart higher education. This essay makes a research proposal for a study using data mining technology to create instructional materials for smart higher education. The analysis of the dynamic scheduling mechanism of intelligent higher education teaching resources based on data analysis technology in unbalanced data environment follows research on the establishment of teaching materials from the discovery of teaching materials, the marking of teaching materials, and the organization of teaching materials. In the end, it is determined that class A students' grades are unquestionably higher than those of class B students. Of course, there are some class B students who score higher than average, but class B students tend to score between 50 and 60 points on average, whereas class A students tend to score higher than average. The contrast is greater, and there are more pupils scoring between 90 and 100. The average grade for students in class A is 80.125, whereas the average grade for students in class B is 71.45. The lowest score in Class B is 51, the lowest score in A is 58, and the greatest score in A is up to 98. It is clear that the development of intelligent teaching resources for higher education based on data mining technology is very successful and has been thoroughly proven.

## 1. Introduction

Teaching resources are an important prerequisite for organizing various teaching tasks [1]. The traditional teaching mode usually spends a lot of manpower and time to organize, compile, and establish relevant teaching resources, in order to ensure the smooth progress of teaching [2]. Traditional teaching resources include paper teaching materials, courseware, electronic teaching images, comprehensive teaching cases, and other teaching resources [3]. Traditional teaching resources lack pertinence in the construction process, and are often only designed for students in specific categories or specialties. When constructing teaching resources, it is necessary to continuously research and analyze teaching objectives, so the educational and teaching resources constructed have better pertinence, and when teaching for a specific teaching group, it will also produce better results.

The use of data is expanding, and more and more people are accumulating a lot of data as human beings get more and more adept at understanding and utilising database technology [4]. The database's tremendous amount of knowledge and data, however, has not yet been fully developed, because the quantity of databases is growing quickly in today's world. Humans must screen the information in the huge data in order to improve screening technology, do better data analysis, and make better decisions [5]. Smart higher education has become an unavoidable trend in the expansion of higher education in the future due to the ongoing reform and growth of the current educational paradigm [6]. The fundamental idea behind smart higher education is to employ information technology to meet students' actual needs, dynamically arrange instructional materials, and carry out corresponding instructional activities in accordance with the demands of various students [7], empowering students to implement rational and scientific instruction in accordance with their knowledge and individual learning capacities in order to reach the goal of overall benefit. The dynamic organization and updating of resources, as well as the dynamic implementation of teaching activities, are given a lot of consideration in the planning and execution of smart higher education. As a result, this article suggests that smart teaching resources for higher education be built using data mining technologies. It provides data support for the creation of a more scientific and objective smart higher education teaching resource through the use of data mining technology and relies on the primary data mining methods, which has some reference significance for the future research on the creation of smart higher education teaching resources.

Data mining is a new, cross-disciplinary field that unites various fields [8]. Data mining is essentially a quick process that involves learning new things. Data mining has currently produced some outcomes [9]. Massive data processing necessitates the use of a complete, intricate, and multidimensional system with numerous data processing modules. In the processed big data system, data mining technology operates as an independent individual, complementing and boosting one another with other modules [10]. Additionally, traditional approaches and techniques for creating instructional resources are no longer able to satisfy the standards of smart higher education. The main determining element is the lengthy and challenging construction cycle of conventional instructional tools. As a result, in accordance with the new smart education model, the conventional approach to planning and creating teaching resources is no longer able to satisfy the current needs of smart education, necessitating a thorough discussion. The use of big data technology to create smart colleges is an unavoidable trend of future development, particularly given the current rapid growth of information technology and computer technology.

The innovation of this paper is that:

1. This paper introduces the current situation of the construction of teaching resources in colleges and universities, and analyzes its design
2. This text research will use data mining technology to obtain comprehensive and in-depth research results on this topic, and promote the construction of smart higher education teaching resources

## 2. Related Work

Data mining is a new technology, it is a new decision support technology, and it is considered to be the most critical step in the database [11]. However, not all information discovery is based on data mining. As a new field of multidisciplinary application, data mining plays an increasingly prominent role in various fields. In most cases, data mining and knowledge discovery in databases are two identical concepts. Data mining is more focused on finding knowledge hidden behind a large amount of data through algorithmic analysis. Data mining technology combines statistics, computer, and other disciplines, can perform data mining on various data, and can perform data mining on structured and unstructured data, which has high practical value.

Liu thinks that the breadth, depth, and subdivision of educational data are all still growing in the big data era. Unstructured, multilayered, and diverse educational data can more accurately and completely describe the educational background and process and outcomes [12]. In the age of big data, Robin noted that students leave a lot of digital traces of their learning processes [13]. Big data, in the opinion of Bachelor, will fundamentally alter modern education in various ways [14]. Big databased learning analysis, according to Cohen et al., can be used to both evaluate courses and teachers and identify and understand the workings of the learning process [15]. Big data technology, according to Dai, has the potential to digitize the entire educational process for kids. The resolution of teaching issues in the big data era will be based on the description and analysis of enormous teaching issues and their solutions [16], rather than on the hazy experience in instructors' brains. Yan and Yang believe that education in the era of big data can break the homogeneity of “one size fits all”; that is, through personalised processing of knowledge transfer, it can better adapt to specific learning environments, students' abilities, and learning preferences [17]. Lee and Cho advocate the use of big data applications in personalised teaching, tailored learning, and personalised engagement because they believe that big data can address the monotonous problem of educational techniques and advance the development of personalised education [18]. Fan and Yang provided a detailed process of data mining service modeling in a cloud environment [19] and presented a data mining service architecture based on cloud computing. Mao et al. use the Apriori algorithm of association rules to analyze the relationship between admission results and candidates' categories and regional grades, allowing education managers to quickly understand the development of education levels in the region and providing more reasonable decisions for the overall arrangement of limited educational resources support [20]. Zhang used the clustering method to reclassify the grades of the four modules of a certain course; then used the association rule algorithm to find the relationship between the categories of departments, the scores of each question, and the total score; and finally used the clustering results and the mined association rules to draw conclusions that are helpful for teaching [21].

The aforementioned researchers have done extensive study on data mining technologies, but creating intelligent teaching tools for higher education requires this technology. Consequently, this study will perform research on the creation of intelligent teaching resources for higher education based on data mining technologies.

## 3. Methodology

### 3.1. Problems Existing in the Current Construction of Teaching Resources in Colleges and Universities

1. Pay close attention to how hardware resources are being built and how software resources are being developed. Many universities have spent a lot of time and money creating networks and buying machinery and equipment, but they have neglected to use the equipment they have acquired, consider how it will affect future resources, and establish application systems, high-quality online resources, and human resources. This is a significant factor in the underutilization of many institutions' campus networks and instructional resources. The purpose of developing teaching resources is the acquisition and sharing of educational resources; network infrastructure is merely a means for information transmission. Building and enhancing campus soft resources is thus a crucial component of creating university campus cultural resources and serves as the foundation for doing so
2. Small quantity, low quality, simple structure, and low efficiency. The construction of network teaching resources should not only digitize and network the traditional teaching resources but also replan, design, and construct based on the characteristics of disciplines and network teaching. The “digital campus” and “online teaching resources” built by many universities are either a simple FTP server or some simple teaching resources, such as exam questions, courseware, web pages, and videos. Single content, general classification, rough production, lack of interaction, inconvenience, and low efficiency. However, some universities' teaching resource library purchases a large number of teaching aids or tapes, and then puts them in the cabinet, causing problems such as difficulty in resource inquiry, low enthusiasm for use, low use efficiency, and poor sharing
3. Lack of standardized teaching resources. The creation of teaching materials is a cumulative process that involves numerous units, people, and resources at various periods. As a result, there is resource content confusion, resource overlap, inconsistent resource nomenclature, format, description, and classification, and inconsistent resource kinds. It is detrimental to management, student learning, and teacher utilization
4. Resource management is simple, inefficient, and lacks security. At present, the storage and management of many educational resources are still in traditional management methods, and have not even been digitalized. Some university management systems have less management, slower update speed, cluttered content, difficult to find, slow speed, difficult to use, ugly interface, and lack of interaction. And many are hacked, security is very low. In this way, teachers and students cannot fully play the role of the resource pool, which leads to a decrease in the utilization rate and actual value of resources
5. Repeated development and purchase of resources. Various universities or the same university, due to the lack of unified coordination, develop, purchase, and construct independently without forming an effective resource sharing mechanism, resulting in a huge waste of human and financial resources
6. Lack of corresponding measures and low enthusiasm for work. Teachers are not motivated, guaranteed, and motivated to design and develop high-quality educational resources, and there is no effective intellectual property protection. Teachers are worried

### 3.2. The Establishment of Teaching Materials

The cornerstone and mainstay of instructional tools are lesson plans. It will eventually become a teaching resource that can accommodate different instructional activities after being collected, sorted, processed, and organized. Therefore, the first issue to be resolved when creating teaching resources is how to gather a big number of teaching materials quickly and effectively. The collection and creation of teaching resources has distinctive qualities in light of the vast computing environment, based on the traditional teaching materials.

Identifying teaching resources: there is a lot of a diversity of different teaching materials available online, and as information technology develops quickly, more and more teaching materials will be released on a regular basis. Online teaching resources are now a highly valuable resource as a result. How to identify instructional resources in such a vast information base is a necessary prerequisite for creating teaching materials. In a large number of resource libraries, use preset relevant teaching materials and some specific keywords to search, analyze, and filter. In addition, there are two main methods for data acquisition: one is to retrieve and analyze a large amount of information through traditional search engines and search tools. The biggest feature of this method of finding textbooks is that it is more maneuverable, but it can only receive some meaningful keywords, so the number and scope of textbooks it can find are very limited. Another method is through automatic search, analysis, and filtering of large amounts of data. Such a search process is more intelligent, and a more intelligent search can be carried out on a larger scale. When constructing teaching resources based on big data, the discovery methods of the two teaching materials can be combined.

The second step is to mark the existing teaching materials. The purpose of labeling teaching materials is to provide convenience for processing and organizing teaching materials in the future, and also to facilitate the organization and use of teaching materials in the future. While labeling teaching materials, it is necessary to organize and transform the found teaching materials, in order to describe, store, and manage according to the unified format set in advance.

The final construction of teaching materials is the unified organization and management of marked teaching materials. Because when organizing and processing teaching resources in the later stage, it is hoped that a very friendly and convenient interface can be used to quickly call and manage various teaching materials. Therefore, it is not enough to describe and annotate only in the form of simple data. The teaching materials are scientifically integrated and organized in order to make better use of these teaching materials in the future. When arranging textbooks, the most important thing is to deal with textbooks of the same type and similar industries. Therefore, there must be a set of professional data organization system to organize textbooks of the same type, different application scopes, and different application fields. In order to organize and process the teaching materials in the future, these materials can be found and organized and processed according to the needs of users.

### 3.3. Construction of Dynamic Scheduling Mechanism for Smart Higher Education Teaching Resources Based on Data Mining Technology

The biggest feature of the teaching resources constructed by smart higher education is to ensure that the educational resources constructed have dynamic variability to meet the dynamic needs of smart higher education. The teaching resources are updated and managed dynamically, and according to these characteristics, comprehensive utilization methods and methods suitable for the changing teaching resources of intelligent higher education are designed. At the same time, a variety of dynamically generated teaching resources can be realized to adapt to the implementation process of intelligent education. According to the research of this paper, the construction of smart higher education teaching resources based on data mining technology, the dynamic scheduling method is mainly implemented in three stages.

1. Data analysis stage: in the data analysis stage, network information will be mined using data mining technology, and the demands of various user groups and users will be analyzed in order to implement teaching activities in colleges and universities. When this technology is used to create teaching resources, users can learn about the many teaching resources that are available on the network by using it. The usage of big data analysis technologies also enables the users to comprehend educational aims and objectives more clearly. It offers solid data backing for the dynamic allocation of teaching resources that follows
2. Demand formation stage. This stage focuses primarily on the distinct teaching objective of intelligent higher education and the method of teaching practice activities, and it calls for the necessary teaching resources. This paper proposes a teaching material discovery and construction mechanism to create a dynamic teaching resource management mechanism to achieve dynamic analysis and management of various teaching materials. It is necessary to conduct a thorough and meticulous analysis of the existing teaching resources when formulating teaching requirements. Learn all there is to know about the current educational materials, then utilise that knowledge to examine the users' instructional needs in great detail and detail. In particular, developing user-related data models and feature models, tracking and analyzing user preferences and characteristics, and creating instructional activities and teaching activities appropriate for students in accordance. On this foundation, dynamic management and the use of the instructional resources in the implementation of the current teaching organization are carried out under the direction of the lesson plan
3. User-oriented teaching resource allocation and management process: this process is unique because it involves the implementation of a teaching organization across a staged and time period. Teachers must repeatedly observe, use, and interact with the process' significant teaching resources. Users can logically organize, integrate, and innovate teaching resources through the integration of teaching resources, particularly through the integration of teaching resources, the integration of teaching resources, and the integration and innovation of teaching resources, and thereby create teaching resources that satisfy users' needs. Finally, the individual requirements of each stage and each process are developed and turned into specialised teaching materials in light of the previously formed specific user needs, directed by the teaching goals of intelligent higher education. It is possible to guarantee the orderly progression of teaching activities at each stage and throughout each process by dynamically allocating the extracted and comprehensive diverse teaching resources. Therefore, it is important to allocate and manage teaching resources in accordance with user demands and characteristics

### 3.4. Data Mining

The method of data mining is shown in Figure 1.

The basic process of data mining is shown in Figure 2. The system use case diagram and structure diagram are shown in Figures 3 and 4. The steps in the process are described as follows:

1. Preparatory stage: this stage involves defining issues, comprehending the corporate objects, gathering data, etc., as well as removing data that is suitable for data mining. It is essential to have a clear grasp of the issue at hand and its intended solution as this will greatly aid in the subsequent evaluation and analysis of the available knowledge. As it takes up nearly half of the overall data mining process, this stage is also the longest
2. Preprocessing: including data cleaning, compression, and transformation. Investigate the quality of the data in order to prepare it for further analysis and determine the type of mining operations
3. Data mining: data mining includes the design and modeling of algorithms. In data mining, how to construct an analytical model suitable for mining algorithms is crucial to the success or failure of data mining
4. Follow-up work: this stage includes interpreting, outputting, evaluating, analyzing and using the results, and interpreting and evaluating the results. The analysis methods it adopts are generally based on data mining operations, and often use visualization techniques

When designing a criterionized database logic, we should also consider properly destroying the criterionized rules. The so-called optimization of data model is to determine the dependence between data and eliminate redundant links in the relational model. In the study, it can be further studied and MSAd by algorithm, as shown in

(1) $$\begin{array}{c} H\left(X\right)=-\overset{R}{\underset{\text{r}=1}{\sum }}p\left(Xi\right)I\left(Xi\right)=-\overset{r}{\underset{r=1}{\sum }}p\left(X\right)\log p\left(X_{i}\right),\\ E\left(E\right)=-\frac{p}{p+N}\log\frac{p}{p+n}-\frac{N}{\text{p}+N}\log\frac{N}{p+N},\\ E\left(E\text{i}\right)=-\frac{pi}{pi+Ni}\log\frac{pi}{pi+ni}-\frac{Ni}{\text{pi}+Ni}\log\frac{Ni}{pi+Ni},\\ E\left(A\right)=\overset{R}{\underset{R=1}{\sum }}\frac{Pi+Ni}{p+N}E\left(Ei\right). \end{array}$$

Therefore, the corresponding algorithm formulas such as formulas (2) and (3) are suggested based on attributes.

(2) $$\begin{array}{c} E\left(Ei\right)=-\overset{c}{\underset{j=1}{\sum }}\frac{P_{ij}}{\left|Ei\right|}\log\frac{P_{ij}}{\left|Ei\right|}, \end{array}$$

(3) $$\begin{array}{c} E\left(A\right)=\overset{v}{\underset{i=1}{\sum }}\frac{\left|Ei\right|}{\left|E\right|}E\left(Ei\right). \end{array}$$

### 3.5. Algorithm Research under Data Mining

#### 3.5.1. Gather Algorithm

With the rapid development of database skill and the diversification of people's means of obtaining data, the amount of data owned by human beings has increased dramatically, but there are few tools for analyzing and processing these data. In recent years, many Gather algorithms have appeared, but none of them can be used to reveal the diverse structure of various multidimensional datasets. The select of Gather algorithm depends on the kind of Gather data, the purpose of Gather, and the applied fields. Because of the intersection of various Gather ways, it is difficult to strictly divide the Gather. The study of data mining way aims to provide the methodology of data mining and formulate the macro strategy to realize the goal of knowledge discovery. Several ways can only solve one data mining problem. Data mining way mainly includes decision tree method, genetic algorithm, neural network method, Bayesian network method, rough set method, rule induction method, database method, and visualization method. In addition, there are fuzzy theory method and information theory method. In the study, the corresponding algorithm formulas are established to MSA and study it, such as

(4) X1∪X2⋯XP=X,Xi∩Xj=f1≤i≠j≤p,dmaxCi,Cj=max∈Ci,p∈C,jp−p dmcanCi,Cj=mi−mj.

Most partition way use distance to describe the similarity between data for Gather. This method can only find spherical classes, but it is difficult to describe any nonspherical classes. Therefore, a density-based Gather method that replaces similarity with density appears. Its main idea is: starting from the distribution density of data objects, connecting the adjacent areas of density, Gather will continue, so that clusters with arbitrary shapes can be found and abnormal data can be effectively handled. This algorithm can not only find any nonspherical class but also effectively filter “noise” data. Density-based Gather algorithm. The advantage of bottom-up grid division method is that it can compress the data into a grid data structure by scanning the data once, so the Gather accuracy obtained is higher, but the computational complexity of the algorithm is larger. In addition, the bottom-up grid method is not suitable for processing high-dimensional data. In recent years, with the emergence of new technologies and ways such as machine learning and artificial mentality, the study of Gather algorithm has become a hot direction in the field of data mining. In decree to improve the ability of large-scale data processing, some scholars have made further study on Gather, and some new Gather algorithm have appeared.

#### 3.5.2. Particle Swarm Optimization

Standard particle swarm optimization algorithm is regarded as the general standard version of the PSO algorithm. The algorithm introduces the inertia coefficient into the basic particle swarm optimization speed update formula *ω* to enhance the space exploration ability of the algorithm and the control of the search range. In the research, the inertia weight *W* decreases linearly from 0.9 to 0.4, and the particle search situation also gradually transitions from the global-based breadth search to the local depth-based search in the process of weight adjustment, realizing the global The balance between search and local search reduces or even eliminates the impact on the performance of the basic particle swarm optimization algorithm when processing the numerical boundary due to the maximum speed. In general, the best global search strategy is to have a good search ability before searching and then get a better seed solution. The so-called breadth search means that the particle will deviate from the original trajectory to find a new solution, while the “depth search” refers to a wider range of accurate search for the current particle near the existing solution.

The particle swarm optimization issue is enhanced in the solution space using both the conventional PSO approach and various upgraded algorithms. If a particle discovers the ideal location during a particle swarm's space search, additional particles will swarm to him right away. The particle swarm will not be able to locate a new global extremum in the solution space if the optimal position is a local rather than a global optimum since the particles will enter a local minimum state. This “premature” technique restricts the particle's search space. The number of swarms must be increased, or the best spots the particles can locate in the current swarm must be weakened, in order to increase the search range. The complexity of the method will increase as the particle population grows, and the particles' pursuit of the global optimum will make convergence challenging. As a result, this research provides a novel particle evolution-based multiparticle swarm optimization technique. The idea of particle evolution is inspired by nature, where the strongest survive. That is, other particles will continue to optimise after a particle enters a local optimum. This method's fundamental principle is to break the group of particles into numerous smaller groups, and the members of each group then adjust the particles in accordance with their individual flight experiences and the “global optimum” of the group to which they belong. When a particle's worst adaptation number reaches a predetermined level, it signals that the particle is no longer appropriate for the current search environment and that an evolution is necessary. During this evolution, the particle's position is reset to the best while the rest of the particles remain in their initial state, continuing this process until all necessary conditions are met. When a person is merely a particle in a group, this particle is referred to as a local version of particle swarm operation. The particle swarm algorithm uses the entire group as a partner.

The basic PSO algorithm and the standard PSO algorithm, both of which are suggested for the optimization of continuous functions, are the discrete examples of algorithms. The continuous domain of the method is based on the continuous domain to optimise the solution. However, a lot of engineering optimization issues, such as combinatorial optimization issues and travelling salesman TSP issues, are based on discrete feature spaces. The fundamental particle swarm optimization algorithm is changed to provide a PSO algorithm suitable for discrete binary version, known as BPSO, in order to more effectively address the discrete optimization problem. Although there are no restrictions on the particle's speed in the discrete PSO algorithm, the value of each dimension in the particle's position vector is only restricted to an integer of 0 or 1. However, the speed is typically used to characterise the integer 0 in each dimension of the position vector or the probability of 1. The likelihood that the corresponding position of the particle will take an integer of 1 is higher if the velocity value of that dimension is larger; conversely, the probability that the corresponding position will take an integer of 0 is higher.

If the mapping function for the particle swarm inertia coefficient is a linear PSO decreasing, the extreme point of the algorithm might not match the extreme point of the actual dynamic system. A larger *ω* PSO will affect *v*_*ij*_ the extreme point where the particle velocity deviates from the current environment. PSO is beneficial to quickly enter the local extremum search, and the extremum of the entire algorithm is better than PSO. Its constraints are

(5) $$\begin{array}{c} 0<\left|v_{i}-\overset{n}{\underset{ii=1}{\sum }}\bar{v_{11}}\right|\ll X\left(d_{m}\right), \end{array}$$

(6) $$\begin{array}{c} H\left(v_{i}\right)=-\overset{n}{\underset{j=1}{\sum }}p_{ij}\ln p_{ij}. \end{array}$$

The particle distance that satisfies the constraints is the *n*′ particle distance in the particle distance pair; then, the average information entropy of particles in the particle distance is

(7) $$\begin{array}{c} \bar{H\left(v_{i}\right)}=-\overset{n}{\underset{j=1}{\sum }}p_{ij}\ln p_{ij}=-\overset{n}{\underset{j=1}{\sum }}\frac{\left|n^{\prime }\right|}{\left|m\right|}\ln\frac{\left|n^{\prime }\right|}{\left|m\right|}. \end{array}$$

#### 3.5.3. Association Rules

The representation of *X*⟶*Y* association *X* rules is called the predecessor in the *Y* association rule and the successor in the association rule. The meaning of *Y* expressions refers to *X* the laws that appear at the same time as they appear.

Item, itemset: An item is an object we study, an itemset is a collection of single or multiple objects, and the objects in the itemset cannot be repeated. Let *I* = {*i*_1_, *i*_2_, *i*_3_, ⋯*i*_*n*_} be an *n* itemset containing items, where *i*_*k*_ is an item and *I* is an *n*− itemset.

Support: Support refers to how often an item occurs in a dataset. The greater the support, the greater the probability that the event will occur.

(8) $$\begin{array}{c} \sup\text{port}\left(A\right)=\frac{\text{count}\left(A\right)}{\text{count}\left(\text{dataset}\right)}=P\left(A\right). \end{array}$$

Confidence: confidence is the number of times; the item*A*coexists with the item*B*, divided by the number of items that only contain the item*A*. It can be understood as*A*the probability that the user buys the product under the premise that he buys the product*B*. The meaning of the confidence is when the confidence is very large, it means that when a user buys*A*, he has a high probability to buy*B*, and then,*A*will make a lot of sense for us to bundle and sell. If the confidence level*B*is very low, it means that when the user purchases*A*and*B*, the probability of purchase is very low; then, this association rule is meaningless. Therefore, confidence reflects whether an association rule can reflect value.

(9) $$\begin{array}{c} \text{confidence}\left(A⟶B\right)=\frac{\text{count}\left(AB\right)}{\text{count}\left(A\right)}=\frac{\text{count}\left(AB\right)/\text{count}\left(\text{dataset}\right)}{\text{count}\left(A\right)/\text{count}\left(\text{dataset}\right)}=\frac{P\left(AB\right)}{P\left(A\right)}=P\left(B\left|A\right.\right). \end{array}$$

## 4. Result Analysis and Discussion

Establish and study data tables for MSA in the study, as shown in Tables 1 and 2.

By constructing the fitness function of its PSO evaluation index system and using the particle mapping PSO candidate teaching resource item set, the dynamic search of the optimal evaluation scheme is carried out under the premise of dimension direction and multiobjective constraints. The experimental simulation shows that the algorithm comparison (as shown in Figure 5) shows that the numerical error of the particle swarm algorithm in this paper is basically within 1, while the other algorithms are within 2. It shows that the algorithm PSO has better evaluation accuracy and execution efficiency.

The convergence accuracy of the algorithm refers to the accuracy calculated by the algorithm when the algorithm runs to the maximum number of iterations. In this PSO, we use the average best test accuracy of multiple experimental test results as a measure. The upper limit of the maximum number of iterations of the function in the PSO test is set to 15. It can be seen from Figure 6 that when the algorithm has a fixed maximum number of iterations, the vector learning PSO learning operator has stronger optimization ability on simple unimodal functions than hybrid learning operators, while on complex unimodal or PSO multimodal functions, the performance of the vector learning operator perturbed by the scalar operator is better. The scalar operator can make the particles escape from the local extreme point through local disturbance, and then can search for a better position. Therefore, in the optimization of multimodal functions, the strategy based on the hybrid operator is relatively better, and its value is basically greater than 1. The maximum value can reach 1.9, and the values of other algorithms are mostly below 3, but we can also see that the Zhongye-discrete learning operator also performs well in the optimization of multimodal functions, and the Zhongye operator can speed up particles The convergence of discrete operators can also make particles avoid local convergence in space search through breadth learning to a certain extent.

Figure 7 shows the results of online random scoring of the teaching construction, due to errors. Therefore, the following is an example analysis of the construction of smart higher education teaching resources based on data mining technology. The study group organized students into two groups, A and B: there were 717 students in group A and 734 students in group B. Thirty-six students were randomly selected to test the satisfaction of two groups A and B on the construction of teaching resources.

Figure 8 shows that the average student results generally follow a similar trend and fall between 50 and 100 points. The two student groups' ratings still differ in a few small ways, though. Most of the students in group A had satisfaction levels that were up to 36 points higher than those in group B, with the majority being higher than 10 points. Some pupils choose to do it the opposite way around. The satisfaction rating for group B is up to 29 points greater than that of group A. Due to the randomness of the students who were chosen at random, they will be split into classes A and B for the investigation.

As can be seen from Figure 9, the overall trend of the average grades of students in the two classes is quite different. The grades of students in class A are obviously better than those in class B. Of course, there are individual students in class B who are more outstanding, but in class B There are more students in the class with a score of 50-60, while the students in class A have more students in the score of 90-100. The contrast is large. The average score of class A students is 80.125, and the average score of class B students is 71.45. The highest score for A can be as high as 98, the lowest score is 58, and the lowest score in class B is 51. It can be seen that the construction of smart higher education teaching resources based on data mining technology is very effective and has been well confirmed.

## 5. Conclusions

In a word, as the application of multimedia technology in the field of education becomes more and more extensive, it will definitely bring about the explosive growth of information resources. Therefore, in the informatization construction of higher education in my country, it is a key issue to build a smart higher education teaching resource construction based on data mining technology. Different from ordinary systems, it involves a wide variety of departments, personnel, and disciplines, complex formats, and great differences in the technical level of operators. Therefore, we should pay attention to the following questions:

1. The high attention of school leaders is a prerequisite for teaching. The leaders of the school have a strong understanding of modern educational technology and educational informatization, have advanced educational modernization and informatization concepts, can increase investment, provide a good informatization environment, formulate policies and reward mechanisms, and establish professional management and information technology. Technical Service Center
2. Organize better and encourage teachers to participate more. In order to raise the level of teaching technology among instructors, the school actively participates in a number of competitions relating to educational information technology held by the educational authorities. In order to enhance students' information technology quality and ability, it is also required to actively participate in education, teaching reform, information technology construction, and the production of high-quality courses, online courses, and courseware
3. The educational technology center and the relevant departments of each school are responsible for technical support and management. The educational technology center should not only provide technical support but also cooperate with relevant departments, such as establishing multimedia technology training for teachers and courseware production, so as to multimedia technology with professional titles and teaching workload
4. Sound security system. The issue of intellectual property rights is an important factor for teachers not to participate in the construction of teaching resource library. Some teachers summed up their experience, accumulated materials, and carefully crafted courseware, which were stolen due to lack of protective measures. To this end, IP restrictions, watermark coverage, PPT, package release, publishing, and other methods should be adopted to solve the intellectual property problems encountered by teachers when sharing resources and to provide teachers with effective services. Only in this way can we ensure the output of high-quality teaching resources and strengthen network security and user review mechanisms to prevent malicious intrusions by hackers
5. Dynamically update teaching resources. In the construction of teaching materials and the discovery of materials, teachers' teaching materials are also constantly increasing and updating. At the same time, the use of these teaching materials to establish teaching resources also needs to be constantly updated dynamically. On the other hand, while implementing intelligent education, the demand for educational resources is constantly changing. Especially in the face of different educational groups and different educational goals, the same teaching content will produce different teaching resources
6. Remote management of teaching resources. Remote monitoring is to allow administrators to remotely view the use and processing of teaching resources. Through remote viewing, users can know which teaching resources are included in the entire teaching resource database, thereby providing the most basic knowledge functions for the subsequent organization and processing of teaching resources. The remote utilization function of teaching resources means that after a user sends a request to a specific resource, the resource can be quickly transmitted to the user's local area, thereby realizing the organization, processing, and application of the resource. Remote utilization is an important means for users to use educational resources for dynamic management. Remote utilization of teaching resources is an important role of users in dynamic management. Its response speed to the user's request and whether the response to the user's request is correct will directly affect the user's experience of the dynamic management mechanism of this teaching resource. The interactive utilization of teaching resources is a relatively complex teaching resource, which can be analyzed, judged, and screened according to the requirements of users, and the required teaching resources can be transferred to the hands of users through a variety of interactive methods. Through multiple interactive data processing processes, the teaching resources that will be finally provided to users can better meet the practical application needs of intelligent higher education, thereby improving the efficiency of teaching resources

## Figures and Tables

**Figure 1:** Main methods of data mining.

**Figure 2:** The basic process of data mining.

**Figure 3:** System use case diagram.

**Figure 4:** System structure diagram.

**Figure 5:** Error comparison chart of the algorithm.

**Figure 6:** Convergence accuracy of algorithm operator.

**Figure 7:** Online random scoring.

**Figure 8:** Group A and group B's ratings of satisfaction with the construction of teaching resources.

**Figure 9:** Grades of class A and class B.

**Table 1:** Data analysis.

Name	Type	Empty	Data
User ID	Int	No	16.62
Username	Varchar	No	25.62
User type	Bit	Yes	53.25

**Table 2:** Data analysis.

Name	Type	Empty	Data
Student card	Int	No	35.63
Student name	Varchar	No	73.62
Sturno	Varchar	No	18.62

## Data Availability

The data used to support the findings of this study are available from the corresponding author upon request.
